# Astaxanthin Enhances Gingival Wound Healing following High Glucose-Induced Oxidative Stress

**DOI:** 10.1155/2022/4043105

**Published:** 2022-03-29

**Authors:** Duru Aras-Tosun, Canan Önder, Nihan Akdoğan, Şivge Kurgan, İrem Aktay, Erkan Tuncay, Kaan Orhan

**Affiliations:** ^1^Department of Basic Medical Sciences, Histology, and Embryology, Faculty of Dentistry, Ankara University, Ankara 06560, Turkey; ^2^Department of Periodontology, Faculty of Dentistry, Ankara University, Ankara 06560, Turkey; ^3^Department of Biophysics, Faculty of Medicine, Ankara University, Ankara 06560, Turkey; ^4^Department of Dentomaxillofacial Radiology, Faculty of Dentistry, Ankara University, Ankara 06560, Turkey

## Abstract

Fibroblasts of the gingiva play a key role in oral wound healing in diabetes. In this study, effects of astaxanthin (ASTX), a xanthophyll carotenoid, were tested on gingival fibroblasts in a wound healing assay in vitro. The aim of this study was to determine whether ASTX can recover delayed wound healing or not when oxidative stress is elevated by high glucose exposure. For this purpose, human gingival fibroblasts were incubated with or without ASTX following exposure to systemic doses of low glucose (LG) and high glucose (HG) in culture media (5- and 25-, 50 mM D-glucose in DMEM Ham's F12) following 24 hours of incubation. Levels of ROS (Reactive oxygen species) were determined for each experimental group by confocal microscopy. Cell proliferation and viability were assessed by an automated cell counter with trypan blue assay. Wound healing assay was designed in 60 mm petri dishes. Cells were exposed to 5-, 25-, and 50 mM glucose for 24 hours, and a straight line free of cells was created upon full confluency. 100 *μ*M ASTX was added to the recovery group, simultaneously. Cells were monitored with JuLI^Ⓡ^-Br Cell History Recorder. ROS levels were significantly increased with increasing glucose levels, while cell proliferation and viability demonstrated a negative correlation with increasing oxidative stress. ROS levels significantly decreased in the 100 *μ*M ASTX-treated group compared to the gingival fibroblasts treated with 50 mM HG medium-only, as well as growth rate and viability. Wound healing was delayed in a dose-dependent manner following high glucose exposure, while ASTX treatment recovered wounded area by 1.16-fold in the 50 mM HG group. Our results demonstrated that ASTX enhances gingival wound healing through its antioxidative properties following high glucose induced oxidative stress. Therefore, ASTX can be suggested as a promising candidate to maintain oral health in chronic wounds of the oral tissues related to diabetes.

## 1. Introduction

Diabetes mellitus (DM) is a chronic, metabolic disease in which blood sugar levels increase due to insulin hormone disorders: one of which is hyperglycemia. Hyperglycemia is responsible for various health complications including cardiovascular diseases, retinopathy, neuropathy, and nephropathy [1, 2], as well as impaired oral health due to increasing incidence of periodontal disease in diabetic patients [3–7].

Chronic inflammation of the periodontal tissues is identified as the periodontal disease [4–8]. In diabetic patients, the course of the periodontal disease may be more severe, as high systemic levels of glucose may contribute to increased inflammation [9] and delayed wound healing via impaired cell migration and proliferation [10–12], increased apoptosis [13, 14], and reduced levels of collagen synthesis [15]. In oral mucosa, gingival fibroblasts play a key role in healing process by production and remodeling of the extracellular matrix (ECM) around the wound tissue [15]. Recently, it has been shown that regeneration capacity of the gingival fibroblasts decreases with increasing concentrations of glucose [16], possibly through a mechanism involving excessive production of reactive oxygen species (ROS) [17].

ROS play a key role in cellular homeostasis via mediation of oxidative stress and inflammation [18, 19]. Low levels of ROS may induce cell cycle arrest, while increased amounts of ROS activate cellular defense mechanisms in vivo. On the other hand, excessive ROS induction is associated with elevated levels of proapoptotic proteins, leading to cell death [20, 21]. Various studies have reported a relationship between oxidative stress and impaired wound healing in chronic, nonhealing wounds due to additional ROS production following prolonged chronic inflammation [22–25]. In diabetic patients with periodontitis, such oxidative damage to cells and tissues of the periodontium is common [22] and has an adverse effect on quality of life [26]. Therefore, reducing the amount of ROS to basal levels is crucial, especially in cases where periodontitis is triggered and/or enhanced by an underlying chronic disease.

On the molecular level, it is possible to prevent these adverse effects through prevention of unwarranted ROS production [27]. Recently, it has been demonstrated that astaxanthin (ASTX), a xanthophyll carotenoid [28], modulates oxidative stress and inflammation through reduction of free radicals [29] and activates endogenous antioxidant systems via genetic modulation [30, 31]. Beneficial effects of ASTX on diabetes, together with or without conventional treatment methods, have been reported [32], including enhanced insulin sensitivity [33, 34], regulation of glucose metabolism [33, 35, 36], and reduction of blood glucose levels [37] in early diabetes, as well as decreased hyperglycemia [37–39], lipid peroxidation, ROS/oxidative stress [40–42], and inflammation [41–45] in diabetes. ASTX is also effective on prevention and treatment of DM-associated pathologies. Positive impact of ASTX has been shown on wound healing in nasal mucosa [46] and vocal fold [47], as well as impaired cutaneous regeneration [48, 49]. However, the effect of the compound on chronic wound healing of the oral mucosa is unknown.

DM is a good model where chronic wound healing is impaired in oral tissues [26]. In this study, an in vitro wound healing assay was designed in gingival fibroblasts following high glucose exposure. The hypothesis tested was that ASTX would reduce levels of ROS induced by high glucose and recover cellular behavior in favor of enhanced wound healing in fibroblasts of the gingiva. Therefore, the aim of this study was to determine whether ASTX can recover delayed wound healing in gingival fibroblasts or not when oxidative stress is elevated.

## 2. Materials and Methods

### 2.1. Cell Culture and Experimental Design

All reagents were purchased from Sigma-Aldrich (St. Louis, MO, USA) unless otherwise stated. Human gingival fibroblasts (Accegen Biotechnology, Fairfield, New Jersey, USA, Cat no: ABC-TC3627) were incubated in low glucose (LG) conditions; in a 1 : 1 mixture of Dulbecco's Modified Eagle's Medium/Nutrient Mixture Ham's F-12 (DMEM/F12) containing 10% heat-inactivated fetal bovine serum (FBS), 100 U/ml-*μ*g/ml penicillin-streptomycin (PS), and 2.5 mg/ml amphotericin B (AMP-B) in a humidified atmosphere of 5% CO_2_ at 37°C. Cells were counted every 24 hours, and number of dead cells was determined with trypan blue assay with an automated device (Vi-Cell, Beckman Coulter, USA). At the end of the 96^th^ hour, *lag* and *log* phases were determined, and population doubling time (PDT) was calculated as explained in Figure 1(a). Total number of live cells was used for the calculation of growth rate.

Culture media was supplemented with D-glucose and/or ASTX for different experimental setups. D-glucose was added to culture media for a final concentration of 25- and 50 mM. ASTX was dissolved in a 1 : 1 mixture of glycerol and culture media as a stock solution. Smaller volumes were dissolved in culture media to obtain a final concentration of 100 *μ*M.

### 2.2. Determination of Intracellular ROS Levels

ROS levels were determined for each experimental group by a Leica TCS SP5 confocal microscope (Mannheim, Germany) equipped with 488 nm argon ion and 543 nm green helium neon laser lines. For this purpose, gingival fibroblasts were loaded with 10 *μ*M of cell-permeant 2′,7′-dichlorodihydrofluorescein diacetate (H2DCFDA; Invitrogen, USA) for 60 min at room temperature (RT), as described previously by Tuncay and Turan [50]. A total of maximum fluorescent intensity from 10 random areas within the range of 30-70 cells were measured following 100 *μ*M H_2_O_2_ exposure and compared to basal fluorescence levels for each cell.

### 2.3. Determination of Cell Proliferation and Viability

Three replicates for each experimental group were treated with either 5-, 25-, or 50 mM D-glucose. Following 24 hours of incubation, an initial number of 0.02 × 10^6^ cells were cultured in 6-well culture dishes. At the 30^th^ hour of incubation (log phase), 100 *μ*M ASTX was added to 50 mM HG-treated cells. Cells were detached from the culture plate with trypsin-EDTA solution (Biochrom, Germany) for 5 min at 37°C, following another 24 hours of culture to determine final number of viable cells. Cell viability was assessed by Vi-Cell as described above.

### 2.4. Monitorization of Wound Healing

Gingival fibroblasts were seeded in standard petri dishes and incubated in LG and HG conditions. When cells reached full confluency, a straight line free of cells was created in the midline with a cell scrapper. 25- and 50 mM HG groups were supplied with D-glucose containing media, while 100 *μ*M ASTX was added to the recovery group, simultaneously. Cells were monitored for an additional 48 hours with JuLI^Ⓡ^-Br Cell History Recorder (NanoEnTek Inc., Waltham, MA, USA) in “Wound Healing” mode in which the confluency of the central scratch was calculated.

### 2.5. Statistical Analysis

Results were shown as mean and standard deviation for three experimental replicates. All statistical analyses were performed with an SPSS software package (SPSS Inc., Chicago, IL, USA). Normally distributed data were analyzed with one-way ANOVA (analysis of variance), and Student's *t*-test was applied to compare groups. The level of significance was *p* < 0.05.

## 3. Results

### 3.1. Effects of High Glucose on ROS Levels

To understand the behavior of gingival fibroblasts in LG conditions, a proliferation assay was performed for 96 hours. PDT was calculated as 29 hours, following a 30-hour *lag* phase (Figure 1(a)). Additional glucose and/or ASTX were added following the *lag* phase in subsequent experiments.

To determine the effects of increasing concentrations of glucose on ROS levels, gingival fibroblasts were incubated in 5-, 25-, and 50 mM glucose containing media. Elevated ROS levels were assessed for individual cells via confocal microscopy. ROS levels were increased in a dose-dependent manner (Figure 2(a)). HG treatment induced oxidative stress significantly in both 25- and 50 mM HG groups when compared to the LG group (*p* < 0.001). Representative confocal images were given in Figure 3 for 5-, 25-, and 50 mM HG groups, respectively.

### 3.2. Effects of High Glucose on Cell Proliferation and Viability

To understand the effects of increasing levels of ROS on cell proliferation, proliferation dynamics of gingival fibroblasts were reevaluated under 25- and 50 mM HG conditions. The LG group was used as a control. Cell proliferation decreased with increasing glucose levels (Figure 1(b)). Growth rate in both 25- and 50 mM HG groups (1.40 ± 0.04 and 1.33 ± 0.1 − fold; *p* = 0.0009 and *p* < 0.0001, respectively) was significantly different than the LG group (1.57 ± 0.04 − fold) (Figure 2(b)).

There was also a negative correlation between ROS levels and cell viability, consistent with the proliferative pattern following HG treatment. The difference between LG (87.67 ± 0.58%) and 25 mM HG groups (83.67 ± 2.31%) was not significant (*p* = 0.1452). Percentage of alive cells was significantly lower in the 50 mM HG group (68.00 ± 6.00%) than the LG group, as well as 25 mM HG group (*p* < 0.001) (Figure 2(c)).

### 3.3. Effects of ASTX on Impaired ROS Levels, Cell Proliferation, and Viability

To determine the protective effect of ASTX on increasing ROS levels, gingival fibroblasts were incubated for 24 hours in 50 mM HG medium suspended with 100 *μ*M ASTX. ROS levels significantly decreased in the 100 *μ*M ASTX-treated group compared to gingival fibroblasts treated with 50 mM HG medium-only (*p* < 0.001). ROS levels were also significantly different in 100 *μ*M ASTX-treated gingival fibroblasts when compared to the LG group (*p* < 0.001). There was no significant difference between the 25 mM HG group and ASTX-treated group (*p* = 0.9432) indicating a remarkable decline in ROS levels of 50 mM HG treated cells following antioxidant uptake (Figure 2(a)).

Impaired cell proliferation and viability was also recovered by ASTX treatment, when compared to the 50 mM HG group (*p* < 0.001). Levels of growth rate were compatible between ASTX- and 25 mM glucose-treated cells (1.43 ± 0.03 and 1.40 ± 0.04 − fold), in line with ROS levels (*p* = 0.2563). There was a significant difference between LG and ASTX-treated groups when number of cells were compared at 24^th^ hour of incubation (*p* = 0.0079) (Figure 2(b)).

### 3.4. Effects of ASTX in Wound Healing

Wound healing was determined with JuLI^Ⓡ^-BR. At 24^th^ hour of incubation, the wound was healed by 96.00 ± 2.65 percent in the control group. The healed area was significantly decreased in both 25- and 50 mM HG groups (85.00 ± 3.00% and 74.33 ± 3.05%; *p* = 0.004 and *p* < 0.001, respectively), while wound healing was enhanced in ASTX-treated cells (86.33 ± 3.05%; *p* = 0.568) responsive to the ROS levels (Figure 2(d)). There was also a significant difference in wound closure when the 50 mM HG and recovery groups were compared (*p* = 0.002) (Figure 4).

## 4. Discussion

Diabetic complications are strongly related to systemic oxidative stress due to high blood glucose levels. One of the most important of these complications is damaged wound closure associated with elevated intracellular ROS [51]. Various in vitro and in vivo studies have confirmed that gingival wound healing is impaired in oral tissues in oxidative stress [52]. Gingival fibroblasts contribute to the regeneration of the gingiva through activation of several genes that have been reported to be involved in tissue remodeling such as control of the cell cycle and proliferation, reorganization of the cytoskeletal proteins, inflammatory response, coagulation, and hemostasis and neoangiogenesis. In this study, an in vitro wound healing model was designed in gingival fibroblasts following high glucose induced oxidative stress. Elevated ROS levels in DM were successfully mimicked in vitro as described previously by Buranasin et al. For this purpose, human gingival fibroblasts were incubated in 5-, 25-, and 50 mM glucose containing culture media for 24 hours. Application of higher doses was not possible due to total detachment of the cells from the culture plate.

Effects of nonsurgical periodontal treatment along with numerous antioxidants have been inspected in clinical studies. Clinical application of coenzyme Q10 and tea tree oil resulted in reduction of clinical markers of chronic periodontitis [53] where vitamin C had no effect on total antioxidant capacity [54]. Short-term efficacy of lycopene was different from long-term treatment [55, 56], together with zinc and selenium [57]. Although therapeutic potential of individual antioxidants such as NAC, taurine and Thai chi were reported in various studies, ASTX was not listed in any clinical studies investigating periodontal regeneration. However, anti-inflammatory and antioxidative effects of ASTX have been reported in various animal models [41, 43, 58]. Zhuge et al. [59] demonstrated that ASTX significantly reduce blood glucose and total cholesterol levels in a dose-dependent manner in diabetic rats. In another animal study by Mizutani et al. [60], it has been demonstrated that insulin resistance is due to oxidative stress impair cell proliferation and angiogenesis in periodontal repair and destruction. Therefore, we have hypothesized that ASTX would reduce levels of ROS induced by high glucose in gingival fibroblasts and enhance wound healing via improvement of cell proliferation and migration.

In this study, ROS was significantly increased with increasing glucose levels, while growth rate and viability of gingival fibroblasts decreased. ASTX treatment recovered ROS levels, enhanced cell proliferation, and decreased cell death significantly. Lately, it has been showed that ASTX reduces increased levels of hyperglycemia-induced ROS production in mitochondria [61] and inhibits inflammation and apoptosis in several tissues and organs [62]. Buranasin et al. have also reported impaired cell proliferation in hyperglycemic gingival fibroblasts, indicating an oxidative stress mediated mechanism in DM patients with delayed periodontal wound healing. In our study, wound healing was delayed in HG conditions compared to the LG group by 1.15-fold, supporting clinical data by Altingoz et al. [63] where different levels of the same oxidative stress markers were reported in diabetic and nondiabetic patients with periodontitis.

Effects of ASTX have been investigated in several wound tissues including nasal mucosa [46], vocal cord [47] and skin [49]. Topical ASTX application reduced ROS production which prohibited inflammatory cell infiltration in epidermis. In the same study, it was stated that wounds treated with ASTX were completely epithelialized on day 9, while the control group showed only partial epithelialization, delaying complete wound closure by two days [48]. ASTX also reduced large amounts of ROS that is produced during vocal fold healing, resulting in decreased tissue contraction and hyaluronic acid deposition [47]. Alongside with protective effects of ASTX, therapeutic effects were also reported in the postinjury period with significantly decreased subepithelial fibrosis. These results suggest that molecular mechanisms of ASTX are not limited to epithelial healing, but also ECM regeneration in vivo.

In our study, protective effect of ASTX in gingival wound healing was demonstrated for both 25- and 50 mM HG exposure. Impaired growth rate and decreased viability were significantly recovered in ASTX-treated group when compared to the 50 mM HG group. Increased cell proliferation and viability, together with enhanced wound closure, was compatible between the 25 mM HG group and ASTX-treated group, but not with the LG group. Higher doses of ASTX treatment did not improve wound healing further (data not shown), indicating necessity of a diabetic animal model for periodontitis to understand the effects of different systemic doses of ASTX in vivo.

## 5. Conclusion

Proliferation and migration of the gingival fibroblasts are crucial for periodontal regeneration. However, hyperglycemia impairs wound healing in gingival fibroblasts due to increasing oxidative stress. In this study, ASTX is suggested as a promising candidate to maintain oral health in DM related wounds of the oral tissue through reduction of oxidative stress.

## Figures and Tables

**Figure 1:** (a) PDT was calculated according to the following formula Tln2/ln (Xe − Xb) (T: time in hours since the beginning of the *log* phase; Xb: number of cells at the beginning of the *log* phase; Xe: number of cells at the end of the total time) as 29 hours and 2 minutes following the lag phase at *t*_30_. (b) Total number of cells at *t*_24_ decreased with increasing glucose concentration. Number of cells was recovered by ASTX application following 50 mM HG treatment.

**Figure 2:** (a) ROS levels were negatively correlated with increasing glucose concentrations, whereas growth rate and cell viability decreased due to intracellular oxidative stress. Oxidative stress in ASTX-treated cells was compatible with the 25 mM HG group, indicating a significant recovery in ROS levels. (b) Growth rate and (c) cell viability were significantly increased following ASTX treatment. (d) Delayed wound healing following increasing ROS levels was recovered following ASTX uptake, due to improved cell proliferation and migration. ^∗∗^*p* < 0.005, ^∗∗∗^*p* < 0.001. Results were shown as mean and standard deviation for three experimental replicates.

**Figure 3:** Effects of ASTX on ROS levels induced by hyperglycemia in human gingival fibroblasts were determined by confocal microscopy. Representative images of DCFDA from 5-, 25-, and 50 mM glucose and ASTX-treated groups are given. To monitor the ROS levels, DCFDA loaded cells were calibrated with 100 *μ*M H_2_O_2_. Changes in total fluorescent intensity in LG group were higher than HG groups, as well as ASTX-treated group (*p* < 0.001). ROS levels were decreased in the ASTX group when compared to the 50 mM HG group (*p* < 0.001). Scale bar: 80 *μ*m.

**Figure 4:** Delayed wound healing in hyperglycemic conditions was impaired following ASTX-treatment. Representative images were from the 24^th^ hour of incubation where confluency was increased by 1.16-fold in ASTX-treated cells compared to the 50 mM HG group (*p* = 0.002). Wounds were closed in both groups at 48^th^ hour.

## Data Availability

The raw data used to support the findings of this study are available from the corresponding author upon request.
